# What Is New in the Preventive and Therapeutic Role of Dairy Products as Nutraceuticals and Functional Foods?

**DOI:** 10.1155/2021/8823222

**Published:** 2021-02-22

**Authors:** Ahmad Taha Khalaf, Yuanyuan Wei, Sadiq Jaafir Aziz Alneamah, Sarmad Ghazi Al-Shawi, Samiah Yasmin Abdul Kadir, Jamaludin Zainol, Xiaoming Liu

**Affiliations:** ^1^Basic Medicine College, Chengdu University, Chengdu, Sichuan 610106, China; ^2^Food Science Department, Agriculture College, Kufa University, Al-Najaf, Iraq; ^3^Food Science Department, Agriculture College, Basrah University, Basrah, Iraq; ^4^Widad University College, 25200 Kuantan, Pahang, Malaysia; ^5^Department of Dermatology, The Third Affiliated Hospital of Southern University of Science and Technology, Shenzhen, China 518055

## Abstract

Nutraceuticals have taken on considerable significance due to their supposed safety and possible nutritional and medicinal effects. Pharmaceutical and dietary companies are conscious of monetary success, which benefits healthier consumers and the altering trends that result in these heart-oriented value-added products being proliferated. Numerous nutraceuticals are claimed to have multiple therapeutic benefits despite advantages, and unwanted effects encompass a lack of substantial evidence. Several common nutraceuticals involve glucosamine, omega-3, Echinacea, cod liver oil, folic acid, ginseng, orange juice supplemented with calcium, and green tea. This review is dedicated to improving the understanding of nutrients based on specific illness indications. It was reported that functional foods contain physiologically active components that confer various health benefits. Studies have shown that some foods and dietary patterns play a major role in the primary prevention of many ailment conditions that lead to putative functional foods being identified. Research and studies are needed to support the possible health benefits of different functional foods that have not yet been clinically validated for the relationships between diet and health. The term “functional foods” may additionally involve health/functional health foods, foods enriched with vitamins/minerals, nutritional improvements, or even conventional medicines.

## 1. Introduction

Functional foods and nutraceuticals play an important role in combating and mitigating diseases and disorders related to lifestyles. These foods contain dietary ingredients that help maintain a healthy lifestyle and can even cure some diseases. Food can be considered functional when it has a significant health effect that extends beyond basic traditional nutrition [1]. Nutraceutical products are derived from foods containing the essential components, like functional foods, which have therapeutic effects. Its beneficial components can be isolated and purified from plant, animal, or marine sources. Functional foods and nutraceuticals have attracted international interest and shaped a growing global market. Often referred to as “functional foods,” nutraceuticals have led to intense controversy due to the fact they blur the conventional dividing line between diet and medicine. Therefore, functional food provides the human body with the required quantity of basic needs and essential for healthy survival like proteins, fats, carbohydrates, and vitamins [2]. It is considered “nutraceutical” when functional food helps in disease/disorder prevention and/or medication other than deficiency conditions such as anemia. Therefore, functional food may be used as a nutraceutical to another consumer. Supplemented dairy foods (for example, milk has a nutrient, and its pharmaceutical product is casein) and citrus fruit (orange juice has a nutrient, and its pharmaceutical constituent is ascorbic acid) are examples of nutraceuticals. This review analyses the fundamental concepts of nutraceuticals and functional foods and discusses some of their sources, including fruits, vegetables, cereals, and legumes [2].

## 2. Nutraceuticals

### 2.1. Concept of Nutraceuticals

Dr. Stephen DeFelice coined the term (nutraceutical) in the year 1989. A hybrid of nutrients and pharmaceuticals underscores the crossroads between the food and pharmaceutical industries. Nutraceuticals contain nontoxic food components that can cure or prevent disease or an unhealthy condition [3]. The concept is by no means new. Almost 2000 years ago, the Greek physician, the father of medicine, Hippocrates said, “Let your food be your medicine and your medicine be your food.” Nutraceuticals play an important role in biological processes like cell proliferation, antioxidant defense, and gene expression. Nutraceuticals can delay the aging process and decrease the risk of situations like cancer, heart disease, hypertension, excessive weight, high cholesterol, diabetes, osteoporosis, arthritis, insomnia, cataracts, constipation, indigestion, and many other lifestyle-related disorders.  Table 1 illustrates the difference between functional foods and nutraceuticals.

Further, nutraceuticals may be isolated and purified from plant, animal, or marine sources. Advantages of nutraceuticals include a longer half-life period, immediate activity upon intake, ready availability, and few side effects. The product soylife helps in the formation of healthy bones, while xangold in maintaining healthy eyes, betatene in immunity improvement, cholestaid and oatwell in blood cholesterol level reduction, and peptopro in the synthesis of muscle protein [4].

The combined and coordinated action of nutrient components and biologically active compounds is flagged as an indication of a “possible beneficial function” to health. Uses and applications of bioactive components cover a wide range of sectors, especially nutraceuticals [5–7]. In vitro [8] and in vivo [9] studies assessing the beneficial effects of nutraceutical models were presented, in particular studies on the nutritional supplements in animals [10–12]. At the same time, particular researches on botanicals have been described by [13–15] concentrating on the importance of those sources of vegetable origin (see Figure 1).

### 2.2. Nutraceutical History

Nutraceuticals are not new to human culture. In fact, they have evolved along with human evolution as a community. Additionally, we learned from experience the health advantages of herbal products; for example, ayurvedic medicines are in the main nutraceuticals, which again suggest their starting point around 5000 BCE and are still commonly used [16].

### 2.3. Nutraceutical Ingredients

Probably any natural, beneficial compounds for both therapy and health, they involved dietary fibers, polyphenols, antioxidants, spices, flavonoids, vitamins, probiotics, and polyunsaturated fatty acids [17]. Believing that functional components will assist in the prevention of diseases leads to a positive attitude towards free fatty acid [18].

### 2.4. Nutraceutical Categorization

Depending on different parameters, many classifications of nutraceuticals were proposed. Depending on the established stage of nutraceuticals [19], nutraceuticals are classified as the following:

1. Nutraceuticals consist of compounds that offer therapeutic benefit in many types of research/epidemiology studies but are lacking compliance with large-scale clinical research
2. Established nutraceuticals consist of compounds that exhibit health benefits well supported by clinical data

They can be divided based on the nutraceutical source from which they are extracted or isolated:

1. Phytochemicals: extracted from plants or herbs such as flavonoids
2. Microbial extracted nutrients: such as vitamin A
3. Nutrients of animal origin: extracted from livestock

Divided based on chemical properties, nutraceuticals are classified as

- Polyunsaturated fatty acids
- Prebiotics
- Flavonoids
- Vitamins

Additional nutraceuticals are classifiable as the following.

1. *Nutritional Enhancements*. These formulas contain nutrients, for example, salt alone or with various preservatives [16].
2. *Functional Foods*. These are defined as food enhanced by promoters who promote optimum health and assist in decreasing the disease risk, such as oatmeal containing soluble fiber that reduces cholesterol levels. They are not just nutrients; in brief, they are foods enhanced with nutrients for health benefits [16].

### 2.5. Nutraceutical Future

Nutraceutical is frequently referred to in the 21st century as a more attractive functional food. By using nutraceutical tools, the physician of the future would have been a better source to offer preventive medical approaches. Nutraceuticals' advances will encourage individualized nutrition personalized to the profile of a person to maximize health and comfort. The nutraceutical market shows that consumers are looking for minimal foods with additional dietary benefits and organoleptic value. In turn, this progress propels the expansion of global nutraceutical markets. In the new millennium, the evolving nutraceutical manufacturing appears destined to occupy the landscape. Its enormous growth and evolution have consequences for food, healthcare, industries of agriculture, and pharmaceutical. As research, exertions continue to unravel the connections between diet and health all over the world. Numerous reviews dealt with the future of nutraceutical markets in the USA, Japan, Europe (pharmaceutical and food opportunities), and Asia (Japan and China) [20].

## 3. Functional Foods

### 3.1. Concept of Functional Food

Functional food is described just like any food or food component that can enhance health beyond fundamental nutrition. Such foods reduce the risk of lifestyle-related disorders by achieving physiological functions beyond nutritional effects. These foods are designed either to prevent or to cure the disease [21]. Specifically, the term “functional food” was created in Japan, which was also the first country to enact legislation that brought functional food products to the market. These foods carry the label Food for Specified Health Uses (FOSHU) in Japan, which underscores the therapeutic focus of these products. Food is made functional in several ways. The functional component is added, removed, or modified during processing or via genetic engineering, resulting in new products that are then introduced into the market. Day et al. have reported that the major challenge for functional foods is to ensure that the bioactive constituents remain stable during processing and storage. Vitamins, fiber, omega-3 fatty acids, minerals, bacterial cultures, and flavonoids are components that can add functionality to any kind of food that is produced [22, 23]. The regular consumption of such foods will help efficiently manage diseases like cardiovascular disease (CVD), tumor, diabetes, and hypertension [24–26].  Table 2 illustrates the various types of common functional foods.

Likewise, many authors have declared about the potential functional foods or their ingredients based on in vitro and animal experiments [27–30], while others misunderstand the difference between conventional and functional foods [31, 32]. Therefore, it is necessary to be aware that functional foods are not medication products, as they do not heal, cure, or prevent diseases (see Figure 2).

### 3.2. Functional Dairy Products

Functional dairy products have undergone an advance as food developed well beyond the fulfillment of the primary needs and were claimed as a treatment aid for primary deficiency syndromes to reduce the risk of disease [33]. Novel yogurt-like products were manufactured using common yogurt starter culture as single or mixed with *Bifidobacterium longum* (ATCC15707) without additives (control) to produce novel functional yogurt-like products [34, 35]. Functional dairy products pose a major challenge to food manufacturing, as the dairy market is already the area where functional foods are more important than incidents and commercial success. Dairy products may be included in the functional food group due to their calcium content, different proteins that improve health, sphingolipids, butyric acid, conjugated linoleic acid, and probiotic cultures [36, 37]. The dairy product industry is well positioned to develop and take advantage of the functional food market [38]. As individuals come to be more health-conscious and more aware of the role nutrition plays in their diets, this opportunity is further enhanced. Consumers want to get further control over their health.

However, the purchaser will now not compromise on taste or product first-class for health products and the rate is a necessary determining factor for repeated purchase. A principal feature of dairy products is that customers already know them, and many accept that dairy products are healthy natural products. Health professionals international inspire a client to eat at various balanced weight loss programs as an alternative than instant solutions being sought, and dairy products are prominent factors for healthy balanced diets. Milk and dairy products make up one of the four predominant groups of meals that form a balanced diet. Moreover, milk is a significant source of protein, B-group vitamins, and calcium in a varied diet and contains vitamin A, thiamine B1, niacin B3, dimethylglycine B16, folate B9, magnesium, and zinc [39]. Marketing “healthy” food has met with market success in the last two decades. Despite the increasing popularity of functional foods, scientists have identified some particular substance or combination of substances that have demonstrated a reduction in disease risk [40, 41]. Furthermore, the addition of a bioactive ingredient to food creates some functional foods. Adding an external ingredient can have an impact on total product acceptance. Many researchers have examined the acceptance by consumers of new functional ingredients of dairy products via using the scale of food neophobia [42], originally suggested by [43]. Gastrointestinal functions are among the most promising aims for functional foods, involving those that control the transit time, intestinal habits, and motility of the intestinal mucosa as well as those that modulate epithelial cell proliferation. Digestive functions are also promising goals related to balanced microflora related to controlling the bioavailability of nutrients, modulating the immune activity of the digestive system, or mediating endocrine activity of the digestive system.

Several systemic functions like lipid homeostasis indirectly influenced by the digestion or fermentation of nutrients are important targets [44, 45]. Darwish has studied the production of functional fermented dairy products using probiotic bacteria isolated from different dairy sources [46]. High-quality empirical evidence research showed that food neophobia is adversely correlated with the willingness of consumers to buy probiotic yogurt. However, this does not affect the willingness of consumers required to purchase other nondairy functional products. Food neophobia with various combinations of functional components can likely play a different role. On the other side, the findings could be complicated by the reality that there is a cholesterol-reducing “virtual prescription” drug for customers with elevated blood cholesterol rates and that therapeutic device developed to reduce neophobia or perception of risk [47] (see Figure 3).

### 3.3. Probiotics in Dairy Products

In recent years, the demand for the use of lactic acid bacteria (LAB) as probiotics has been growing. In addition to acid and bile resistance, the key trait for a LAB strain to be a probiotic is the capacity to generate antimicrobial compounds in opposition to pathogenic and cariogenic bacteria and to bind to and colonize the intestinal mucosa of humans. Moreover, the development of antimicrobial compounds supports the colonization of probiotics in intestine mucosa via raising their competitive benefit over normal gastrointestinal microflora. Research has proven that capsular polysaccharides could encourage adherence of bacteria to biological surfaces and, thus, facilitate the colonization of different ecological niches [48]. Many of the health benefits of probiotics consist of stimulating immunity, playing an adjunctive role to a vaccine, adhering to cells in the human gut, and increasing aiding in the production of vitamin K and vitamin B, as well as strengthening the protective barrier of the digestive system and preventing diarrhea caused by radiation therapy as antibiotics for rotavirus and C. Furthermore, it is effective in the treatment of constipation, prevention of inflammatory intestinal disorders, and anticancer action, as well as reduces blood pressure and lowers cholesterol [49]. Research has revealed that certain lactobacilli strains have antioxidant activity and may decrease the risk of accumulation of free radicals [50]. Furthermore, probiotics modulate inflammatory and hypersensitivity responses. This may be because of cytokine function regulation. They prohibit reoccurrences of inflammatory intestinal disorder in adults as well as improved milk allergies and reduce children's eczema risk. Probiotics improve the allocation of immune function by increasing the number of plasma cells developing IgA, increasing or enhancing phagocytosis, and raising the ratio of natural killer cells and T lymphocytes [51]. Due to the production of the Angiotensin-Converting Enzyme (ACE) inhibitors, such as peptides during fermentation, the intake of fermented milk with different LAB strains can lead to moderate blood pressure reductions [52].

In animals, lowering the serum cholesterol levels through probiotics can presumably be achieved by decomposing bile in the intestines, thereby preventing its reabsorption. This can lead to modest reductions in total cholesterol and LDL levels [53]. Most probiotics have been used for GIT-related diseases; however, some studies have probiotics assessed in allergic conditions, along with dermatitis, rhinitis, vaginosis, and allergies to foodstuffs. Atopic dermatitis, known as eczema, is the most popular of skin disorders. Studies have proven that probiotics, such as *Lactobacillus rhamnosus* GG, may forestall or decrease the symptoms. In addition, eczema can be avoided if moms eat probiotics for the duration of their pregnancy and if neonates consume it during the first six months of their existence [54]. Probiotics like *Lactococcus*, *Leuconostoc*, and Pediococcus can prohibit or restrict cycotoxinogenic mildew increase [55]. Besides, LAB could bind aflatoxin B1 both in vivo and in vitro according to their bacterial strain [56]. Previous studies suggested that *Lactobacillus paracasei* reduces body and belly fat. Apparently, these probiotics have an antiobesity effect [57]. Most possibly, intestinal bacteria can control body weight by influencing the metabolic neuroendocrine and immune functions of the host [56].

### 3.4. Probiotic Yogurt as a Functional Food

Yogurt is a result of milk fermentation with lactic acid by adding a common starter culture that includes *Streptococcus thermophilus* and *Lactobacillus delbrueckii ssp. bulgaricus*. Less typical microorganisms in some countries, like *Lactobacillus delbrueckii ssp. lactis* and *Lactobacillus helveticus*, often mixed with a mixture of starters [58]. Currently, the market provides a wide range of yogurts suitable for all palates and meal occasions. Yogurts come in a diversity of textures (like liquid, stirred, and set), flavors (like natural, fruit, and cereal), and fat contents (like luxury, low-fat, and fat-free); can be enjoyed like a snack or as part of a meal, like sweet or savory snacks; and are available throughout the year. Together with their recognition as healthy and nutritious food, this versatility contributed to their widespread success in all subgroups of the population. Introducing probiotic strains to yogurt is a good approach to produce effective, acceptable, and affordable fermented milk. However, introducing new strains to yogurt starter culture may affect the acidity, aroma perceptions, and textural properties of the product. The texture is a critical aspect of yogurt that is acceptable to consumers. Rheological properties affect the texture that affects sensory perception and ultimately consumer acceptance of a product [59–61]. Functional properties of microorganisms in fermented foods contain probiotics [62], antioxidants [63], antimicrobials [64], peptide production [65], polyglutamic acid [66], fibrinolytic activity [67], and antinutritional compound degradation [68]. Proteolytic microorganisms through food fermentation [65], which exhibits certain functional properties like immunomodulatory properties [69], antihypertensive properties [70], and antithrombic properties [71], form bioactive peptides.

### 3.5. Health Benefits of Functional Foods

Marco et al. described that enhanced nutritional and functional properties of fermented foods maybe because of the transformation of substrates and formation of bioactive or bioavailable end products [72], while Sarkar confirmed the most promising targets of functional foods as [73]

- intestinal function including those control transit time, bowel habits, mucosal motility, and modulation of epithelial cell proliferation
- gastrointestinal (GI) function that is associated with a balanced colonic microflora, control of nutrient bioavailability, and modification of GI immune activity or that is mediated by the endocrine activity of the GI system
- systemic function such as lipid homeostasis that is indirectly influenced by the nutrient dosage or fermentation

Further, he also highlighted the extension of the following health benefits to human beings due to the consumption of functional foods [73]:

- Reduced risk of cardiovascular disease
- Reduced risk of cancer
- Improved health in general
- Improved memory
- Improved weight loss/management
- Reduced risk of other diseases
- Reduced osteoporosis
- Improved mental health
- Quicker reaction time
- Improved fetal health

### 3.6. Health Benefits of Nutraceuticals

Nutraceuticals are used in an attempt to accomplish desirable therapeutic outcomes with reduced side effects, as compared with other therapeutic agents. Consumption of plant-based foods, nuts, whole grains, cereals, and marine foods plays a vital role in disease prevention and health promotion [74, 75]. Some popular nutraceuticals include lutein (for macular degeneration), folic acid, and cod liver oil capsules. The most popular functional food and beverage products include omega-3 eggs, omega-3-enriched yogurts, calcium-enriched orange juice, and green tea, to mention a few.

The majority of the nutraceuticals do possess multiple therapeutic benefits. Nutraceuticals are claimed to possess physiological benefit or protection (Figure 4) against the following diseases:

- CVD
- Cancer
- Diabetes
- Obesity
- Chronic inflammatory disorders
- Parkinson's disease
- Alzheimer's disease

## 4. Conclusion

The goal of this article is to encourage medical and health professionals to expand their knowledge of the properties of functional foods as they promote good health while helping to prevent disease. Functional foods that contain physiologically active ingredients can improve health, from either animal or plant sources; by supporting health through prevention rather than treatment, nutraceuticals and functional foods could provide a solution to reduce the growing burden on health care systems, although it is important to note that functional foods are not medications, as they do not heal, cure, or prevent diseases. However, nutraceutical products are expected to play a major role in potential therapeutic development. Society health authorities regard nutraceutical as prevention, therapy, and a powerful tool for preserving health and acting versus acute and chronic diseases caused by nutrition, thereby enhancing health. Nutraceuticals are developing in clinical practice, but advanced studies need to address the importance of pharmaceutical and clinical issues.

## Figures and Tables

**Figure 1:** Concept of nutraceuticals [15].

**Figure 2:** Establishing functional foods [32].

**Figure 3:** Dairy products.

**Figure 4:** Nutraceuticals used in prevention of various diseases [74].

**Table 1:** Difference between functional foods and nutrients with examples.

Functional foods	Nutraceuticals
The foods with ingredients which give that food health-promoting properties over and above its usual nutritional value	The foodstuff (as a fortified food or a dietary supplement) held to provide health or medical benefits in addition to its basic nutritional value
Naturally contain bioactive compounds found in foods	The bioactive compounds found in fortified foods, dietary supplement, or herbal products
Natural	Natural or synthetic and available as pills, capsules, or liquids
The bioactive compounds in them are different from the traditional nutrients	Include traditional nutrients
Grapes, strawberries, and apple are examples	Beta-carotene, lycopene, resveratrol, and ferulic acid are examples

Source: Mulry [4].

**Table 2:** Various types of functional foods.

Type	Description	Example

Enriched food products	Adding new nutrients or ingredients that are not usually found in food	Fruit juice enriched with calcium, foods with probiotics and prebiotics

Enhanced food commodities	Changes in raw materials that altered the nutrient composition	Carotenoid-containing potatoes, high-lysine corn

Fortified food products	Increase the content of nutrients present	Grain products fortified with folic acid, fruit juice with extra VC

Altered food products	Change existing components with beneficial components	Low-fat foods with fat replacers

Source: Spence [27].
